This article has been retracted.

# Combined effect of Zinc lysine and biochar on growth and physiology of wheat (*Triticum aestivum* L.) to alleviate salinity stress

**DOI:** 10.3389/fpls.2022.1017282

**Published:** 2023-03-09

**Authors:** Zain ul Aibdin, Muhammad Nafees, Muhammad Rizwan, Shoaib Ahmad, Shafaqat Ali, Wael A. Obaid, Moodi Saham Alsubeie, Doaa Bahaa Eldin Darwish, Amany H. A. Abeed

**Affiliations:** ^1^ Department of Environmental Sciences, Government College University Faisalabad, Faisalabad, Punjab, Pakistan; ^2^ State Key Laboratory of Pollution Control and Resource Reuse, School of the Environment, Nanjing University, Nanjing, Jiangsu, China; ^3^ Department of Biological Sciences and Technology, China Medical University, Taichung, Taiwan; ^4^ Department of Biology, College of Science, Taibah University, Al-Madinah Al-Munawarah, Saudi Arabia; ^5^ Biology Department, College of Science, Imam Mohammad Ibn Saud Islamic University (IMSIU), Riyadh, Saudi Arabia; ^6^ Department of Biology, Faculty of Science, University of Tabuk, Tabuk, Saudi Arabia; ^7^ Botany Department, Faculty of Science, Mansoura University, Mansoura, Egypt; ^8^ Department of Botany and Microbiology, Faculty of Science, Assiut University, Assiut, Egypt

**Keywords:** saline soil, wheat, biochar, zinc lysin, antioxidants, nutrient contents

## Abstract

Globally, Food security main threaten by abiotic stress like salinity and levels amongst the majority serious environmental stressors which reduce crop yield mass production. Biochar application has received much attention in agricultural practices as it enhances crop quality and production. The present study was carried out to analyze the role of lysine zinc and biochar on growth enhancement of wheat (*Triticum aestivum* L. cv. PU-2011) under saline stress (EC 7.17 dSm^-1^). Seeds were sown in pots containing saline soil with and without 2% biochar, and foliar application of Zn-lysine (0, 1.0, and 2.0 mM) was made at different time intervals during plant growth. A combined application of biochar and Zn-lysine 2.0 mM highly improved the physiological attributes such as chlorophyll a (37%), chlorophyll b (60%), total chlorophyll (37%), carotenoids (16%), photosynthesis rate (*Pn*) 45%, stomatal conductance (*gs*) 53%, transpiration rate (*Tr*) 56%, and water use efficiency (*WUE*) 55%. The levels of malondialdehyde (MDA) 38%, hydrogen peroxide (H_2_O_2_) 62%, and electrolyte leakage (EL) 48% were decreased with the combined application of biochar and Zn-lysine 2.0 mM as compared with other treatments. The activities of catalase (CAT) 67%, superoxide dismutase (SOD) 70%, and ascorbate peroxidase (APX) 61% as well as catalase (CAT) 67% were regulated with the combined biochar and Zn-lysine 2.0 mM treatment. Similarly, the combined application of biochar and zinc-lysine (2.0 mM) enhanced the growth and yield attributes such as shoot length (79%), root fresh weight (62%), shoot fresh weight (36%), root dry weight (86%), shoot dry weight (39%), grain weight (57%), and spike length (43%) as compared with untreated control. The concentrations of sodium (Na) decreased whereas potassium (K), iron (Fe), and zinc (Zn) concentrations were enhanced in plants with the combined application of Zn-lysine and biochar. Overall, results showed that the combined application of Zn-lysine (2.0 mM) and biochar significantly inhibited the negative effect of salinity and improved the growth and physiological performance of wheat plants. The combined use of Zn-lysine and biochar might be a practical solution to tackle salt stress in plants, but field studies by growing various crops under varied environmental conditions are needed before any recommendation to farmers.

## Highlights

➢ Salinity stress significantly reduce the physiological attributes and growth of wheat
➢ Zn-lysine (2.0 mM) and biochar alone and in combination enhanced the biomass of wheat
➢ Zn-lysine and biochar alone and in combination improved the antioxidant activity in leaves under salt stress
➢ Zn-lysine (2.0 mM) and biochar assisted the nutrient uptake by wheat plants under salt stress.

## Introduction

In developing countries, Agriculture is the economic backbone and main source of income for the countryside people (Mishra et al., 2014). The primary origin of food is the agriculture, and it is anticipated to feed an ever-growing global population through improving agricultural practices (FAO, 2014). Wheat (*Triticum aestivum* L.) is an important staple meal for 4.5 billion public people around the world, which is providing about 20% of their daily protein and calories (Foley et al., 2011). Wheat demand is predicted to reach 536 to 551 million tons within a decade as a result of sustained human population growth (Van Bavel, 2013). Wheat is a popular food crop because of its flavor and nutritional value such as calories, proteins, and vitamins (Ahmad et al., 2022). Wheat and flour-milling by-products of poor grade are utilized as livestock feed. Plants require micronutrients for the growth and regulation of critical physiological functions, although micronutrients are required in small amounts but are just as significant as macronutrients for plant growth and proper functions. Micronutrient deficiency in Pakistan is caused by calcareous soils, high pH, poor soil organic matter, salt stress, and use of unbalanced NPK fertilizers along with other factors. Salinity is the major abiotic stress affecting agricultural land throughout the world (Ali et al., 2017; Saifullah et al., 2018). Globally, approximately 1,128 M ha of agricultural fields have been spoiled due to salinity and sodification (Wicke et al., 2011). Soil salinity which is primarily caused by excess soluble salts in agricultural fields is one of the most serious risks to crop productivity especially cereals such as wheat. At high salinity levels, the concentration of sodium ions (Na^+^) may cause changes in soil physicochemical features such as decreased soil porosity, infiltration, aggregate stability, aeration, and water conductivity which may impair the plant nutrient uptake availability and overall soil health (Adnan et al., 2022). Among cereals, wheat productivity is seriously affected due to excess salt stress (Ali et al., 2017). Salinity has shown negative effects on wheat growth parameters such as panicle initiation, number of tillers, spikelet formation, grain size, delayed heading, and physiological features (Negrao et al., 2017). Thus, salt stress needs to be addressed on an urgent basis to avoid reduction in wheat growth, which is much needed to feed the ever-increasing world population.

The usage of micronutrients may be effective in decreasing detrimental effects of abiotic stresses in plants (Bashir et al., 2018). Salt stress in plants might be addressed by providing suitable nutrients to the plants especially micronutrients such as zinc (Zn). Zinc is a micronutrient that is necessary for healthy growth and development of plants (Rizwan et al., 2017). Appropriate Zn content in seeds improves seed germination under less-than-ideal conditions, viability, and stand establishment. High level of pH, salinity, calcium, and bicarbonates; waterlogging; intense farming; and increased nutrient consumption are all associated with Zn shortage in soil (Alloway, 2008; Alloway, 2009). Fertilizers such as amino acids and iron (Fe) as well as Zn like lysine, were demonstrated to improve the yield development and growth of the crop (Souri, 2016; Rafie et al., 2017). Supplementing plants with zinc–lysine significantly improved plant growth, photosynthesis, and nutrient contents in plants (Rizwan et al., 2017; Noman et al., 2018). Zn chelated with lysine enhanced the chlorophyll contents and gas exchange attributes in leaves by improving plant nutrition (Ghasemi et al., 2012). The studies reported the positive effects of Zn–lysine in alleviation of heavy metal toxicities in plants (Rizwan et al., 2017; Hussain et al., 2018). However, the effects of Zn–lysine to alleviate salt stress in plants need to be explored. In addition, less is known about the effects of Zn–lysine combined with other suitable amendments under abiotic stresses in plants.

Biochar, Material like a charcoal a is being more widely utilized in agriculture to improve soil fertility, increase crop yield, trap carbon in the soil, and reduce greenhouse gas emissions (Lehmann, 2007; Pan et al., 2009; Zhang et al., 2010; Cayuela et al., 2013; Abiven et al., 2014). Pyrolysis is a method that involves warming the agricultural residue animal or poultry manures at high temperature. Because of its strong aromaticity, it is quite recalcitrant in nature (Keith et al., 2011; Singh et al., 2012; Zimmermann et al., 2012; Fang et al., 2014; Kuzyakov et al., 2014). Recently, biochar utilization in agriculture received much attention as a soil amendment. Biochar has potential to increase crop production by enhancing the soil physical, chemical, and biological properties such as aggregate stability, porosity, saturated hydraulic conductivity, water holding capacity, bulk density and particle density, nutrient retention, cation exchange capacity (CEC), EC, and pH, microbial population in the rhizosphere, microbial biomass C and N, and enzymatic activity (Lehmann and Joseph, 2009; Sohi et al., 2010). Biochar has magic properties to adsorb salts and other elements present in the soil (Thomas et al., 2013; Abbas et al., 2017). In a study, Parkash and Singh (2020) showed that biochar application enhanced the stomatal conductance and photosynthesis and decreased the leaf temperature and electrolyte leakage in eggplant leaves. Previous studies showed that biochar alleviated the salinity stress and increased the growth and production of potato and wheat (Akhtar et al., 2015a; Akhtar et al., 2015b). Although biochar is effective in minimization of abiotic stresses in plants, the role of biochar along with Zn–lysine is not studied under salt stress in plants.

In this study, it has been hypothesized that under the salt stress by applying the combine application of biochar and Zn-lysine may enhance the growth of wheat crop by alleviating the negative effect of salinity in plants. The objective of the present study was to explore the morph-physiological response, photosynthesis, selected nutrients (potassium, phosphorus, iron, Zn), and Na uptake by wheat under salt stress treated with foliar applied Zn–lysine alone or combined with soil applied biochar. This study will offer new insights into the application of Zn–lysine and biochar to cope with salinity stress in wheat and probably other crop pants.

## Materials and methods

### Soil analysis and collection 

This experiment was conducted in the soil collected from the field of Ayub Agriculture Research Institute located in Pakka Anna village, Toba Tek Singh, Punjab, Pakistan. Soil was mildly saline with an EC of 7.17 dSm^-1^. Soil was sieved through a 2.0-mm sieve to remove roots and debris present in the soil. The standard protocols were employed to analyze the particle size, pH, and EC of the soil (Bouyoucos, 1962). After treating soil with an AB-DTPA solution at pH 7.6, the available trace elements were determined (Soltanpour, 1985). The Walkley–Black method (Jackson, 1962) was employed to determine soil organic matter, whereas the calcimeter method was utilized to estimate calcium carbonate (Moodie, 1959). Soil is saline in nature; the selected soil initial properties are described in **Table 1**.

**Table 1:** Physicochemical properties of soil.

Soil	Unit
**Textural Class**	Sandy Clay Loam
Sand	63.7%
Silt	14.4%
Clay	21.9%
**Saturation percentage**	30%
pH	7.71
EC	7.17 dSm^-1^
HCO_3_	(7.15 mill mole L^-1^)
Total nitrogen	0.07%
Available P	6.32 ppm
Extractable K	290 ppm
Ca^+2^ + Mg^+2^	(14.92 mill mole L^-1^)
Rice husk Biochar	
pH	8.85
EC	3.1 dSm^-1^

### Preparation of biochar

Biochar was made from rice husks as a feedstock by using furnace manually prepared for biochar production in which indirect heat was provided to the feedstock, and biochar was prepared under a limited oxygen environment. Slow pyrolysis was done with a gradual increase in temperature, and a final temperature of 400°C was maintained for 3 h to pyrolyze the rice husk. The biochar was analyzed for EC and pH which were determined using a suspension (1:10 w/v) and standard buffer solutions using a pH meter with gloss electrodes, and EC was determined using a conductivity meter according to the techniques specified by Rowell (1994); data are reported in **Table 1**.

### Treatments and experimental design

The pot experiment was carried out in the botanical garden of Government College University, Faisalabad-Pakistan, in natural environmental conditions with a 27/21°C (day/night) temperature range at the time of sowing (**Figure 1** schematic diagram). Furthermore, the average humidity during the experiment was 68%. Plastic pots were filled with sieved soil (5 kg pot^-1^), and biochar (2% w/w) was added in half of the pots; all the pots were treated with foliar spray of Zn–lysine (0, 1.0, and 2.0 mM) during the plant growth (after 2 weeks of germination) in triplicate using a completely randomized design (CRD). In each pot, eight seeds of bread wheat (variety Punjab-2011) were planted. Following germination, thinning was done, and four healthy plants were left in each pot. Pots were irrigated using good-quality tap water (1.12 dSm^-1^) to control salinity stress during the entire growth duration.

**Figure 1:** Data represent different levels of zinc–lysine (control 0, 1, 2 mM) with and without biochar on chlorophyll a, chlorophyll b, total chlorophyll, carotenoid, *Pn*, *gs*, *Tr*, and *WUE* contents of wheat plant showing means of replicates (n = 3) ± standard deviation. Different letters indicate significant differences by Tukey HSD test at *p* ≤ 0.05.

### Harvesting

Plants were collected 4 months after seeding. After measuring wheat plant height and spike length, the plants were divided into shoots, roots, spikes, and grains. Roots were cleaned with double d-H_2_O before being cleaned with dilute hydrochloric acid (0.1% HCl). The dry weights of oven-dried roots and shoots (72 h at 70°C) were determined, and the dried samples (root, shoot, and grains) were ground into powder for further analysis.

### Physiological attributes

Physiological attributes were determined when the plants were 90 days old through apply portable infrared gas analyzer (IRGA) on a sunny day about (10:00–12:00 a.m.). Fully extended plant leaves from each pot were chosen to measure the value of *gs*, *Tr*, *WUE*, and *Pn*. Healthy and fresh leaves from plants were selected to assess the photosynthetic pigments, i.e., total chlorophyll, chlorophyll a, b, and carotenoids (Lichtenthaler, 1987). To assess the chlorophyll and carotenoid concentrations, samples were processed in 85% acetone (v/v ratio) and centrifuged, and readings were taken at specified wavelengths using a spectrophotometer.

### Malondialdehyde, electrolyte leakage, hydrogen peroxide, and antioxidant enzymes

MDA levels were determined using 0.1% thiobarbituric acid (TBA) Zhang and Kirham (1994). Dionisio-Sese and Tobita’s (1998) technique was used to estimate EL. Measurement was done in two steps: first, plant leaf samples have been extracted at 32°C for 2 h to obtain the initial reading of EC of the samples, then samples have been heated on a water bath at 121°C for 20 min to obtain the final reading of EC.

EL = (EC1/EC2) 100

The contents of H_2_O_2_ were calculated using the procedure of Jana and Choudhuri (1982). These samples were homogenized before centrifugation by addition of phosphate buffer (50 mm at pH 6.5) followed by 20 min of centrifugation. Afterward, H_2_SO_4_ (20%, v/v) was added to the ultra-spin extract followed by another 15-min centrifugation. At a wavelength of 410 nm, the absorbance was measured. Samples were homogenized in phosphate buffer (0.5M at pH 7.8) to determine POD and SOD activities (Zhang et al., 1992). The activity of APX was measured using the Nakano and Asada (1981) procedure, and CAT activity was calculated following Aebi’s (1984) method.

### Growth attributes and biomass

Plant shoot lengths (cm) were recorded by using a measuring scale, fresh and dry weight of shoots and roots (g per pot) by a weight balance, the length of spike (cm) by a measuring scale, and grain weight (g) by using a weight balance; all these were measured as growth characteristics.

### Metal contents in plants

Fe, K, Zn, and Na concentrations were analyzed in roots, shoots, and grain samples. The plant samples were digested using diacid digestion (HNO_3_: HClO_4_; 4:1 v/v). Digested samples were diluted, and nutrient Fe, K, Zn, and Na concentrations in plant parts (mg kg^-1^ of dry weight) were determined using an atomic absorption spectrophotometer (AAS) for detection of metals (Rehman et al., 2015). P concentrations in plant tissues were measured by the procedure of Ohno and Zibilske (1991).

### Data analysis

The IBM SPSS (Version 21.0) software for Windows was used for the statistical analyses. Analysis of variance (ANOVA) was applied using complete randomized design at a significant ≤5% probability level. Tukey’s HSD *post-hoc* test was applied for multiple comparisons of means.

## Results

### Physiological attributes

The highest plant physiological attributes were found with the combined application of zinc–lysine (2.0 mM) and biochar. Similarly, physiological attributes such as chlorophyll a, b, total chlorophyll, carotenoids, *Pn*, *gs*, *Tr*, and *WUE* were increased with the combined application of zinc–lysine (2.0 mM) and biochar, as shown in **Figure 2**, whereas chlorophyll a (24%), chlorophyll b (36%), total chlorophyll (23%), carotenoids (3%), *Pn* (30%), *gs* (44%), *Tr* (29%), and *WUE* (37%) were increased with zinc–lysine (2.0 mM) alone treatment as compared with control, and chlorophyll a (37%), chlorophyll b (60%), total chlorophyll (37%), carotenoids (16%), *Pn* (45%), *gs* (53%), *Tr* (56%), and *WUE* (55%) were increased with the combined application of zinc–lysine (2.0 mM) and biochar as compared with control (**Figure 2**).

**Figure 2:** Data represent different levels of zinc–lysine (control 0, 1, 2 mM) with and without biochar on MDA, H_2_O_2_, EL, POD, SOD, APX, and CAT contents of wheat plant showing means of replicates (n=3) ± standard deviation. Different letters indicate significant differences by Tukey HSD test at *p* ≤ 0.05.

### Oxidative stress and antioxidant enzyme activities

Oxidant (MDA, H_2_O_2_, EL) and antioxidant enzymatic activities (POD, SOD, APX, and CAT) in leaves of wheat plants were measured; data are shown in **Figure 3**. MDA, H_2_O_2_, and EL were statistically higher under salt stress. Similarly, POD, SOD, APX, and CAT activities were increased due to activation of the defense mechanism under salt stress. The application of zinc–lysine (2.0 mM) decreased MDA, H_2_O_2_, and EL (30%, 60%, and 34%, respectively) as compared with control treatment, whereas the highest reduction in MDA (38%), H_2_O_2_ (62%), and EL (48%) was observed with the combined application of zinc–lysine (2.0 mM) and biochar as compared with control (**Figure 3**). On the other hand, the application of zinc–lysine (2.0 mM) statistically enhanced the POD (16%), SOD (35%), APX (36%), and CAT (26%) activities in leaves under salt stress compared with control treatment. Similarly, the combined application of zinc–lysine (2.0 mM) and biochar further increased the POD (44%), SOD (70%), APX (61%), and CAT (67%) activities as compared with control (**Figure 3**).

**Figure 3:** Data represent different levels of zinc–lysine (control 0, 1, 2 mM) with and without biochar on shoot length, shoot fresh weight, shoot dry weight, root fresh weight, root dry weight, grain weight, and spike length of wheat plant showing means of replicates (n = 3) ± standard deviation. Different letters indicate significant differences by Tukey HSD test at *p* ≤ 0.05.

### Growth parameters

It was observed that the salinity stress drastically decreased the shoot length, root and shoot fresh and dry weights, grain weight, and spike length as compared with the alone and combined application of biochar and zinc–lysine (1.0 and 2.0 mM), as shown in **Figure 4**. Zinc–lysine (2.0 mM) increased the shoot length (50%), root fresh weight (34%), shoot fresh weight (17%), root dry weight (49%), shoot dry weight (16%), grain weight (28%), and spike length (25%) as compared with control treatment. Similarly, the combined application of zinc–lysine (2.0 mM) and biochar significantly enhanced the shoot length (79%), root fresh weight (62%), shoot fresh weight (36%), root dry weight (86%), shoot dry weight (39%), grain weight (57%), and spike length (43%) as compared with untreated control (**Figure 4**). The combined application of zinc–lysine (2.0 mM) and biochar on yield components resulted in higher grain weight which ultimately indicated a higher number of spikes per plant and a higher number of grains per spike.

**Figure 4:** Data represent different levels of zinc–lysine (control 0, 1, 2 mM) with and without biochar on P in shoot, P in root, Fe in root, Fe in shoot, K in root, K in shoot, Na in root, Na in shoot, Zn in root, Zn in shoot, Zn in grain, and Na in grain of wheat plant showing means of replicates (n = 3) ± standard deviation. Different letters indicate significant differences by Tukey HSD test at *p* ≤ 0.05.

### Nutrient uptake

The concentrations of P, Fe, K, Na, and Zn were measured in different parts of wheat; data are reported in **Figure 5**. Results showed that the application of zinc–lysine (2.0 mM) enhanced the P (21% and 19%), Fe (39% and 23%), K (24% and 47%), and Zn (106% and 163%) contents in roots and shoots, respectively, as compared with control, whereas the fortification of zinc–lysine (2.0 mM) decreased the Na content (52% and 46%) in roots and shoots, respectively, as compared with control. Similarly, the combined application of zinc–lysine (2mM) and biochar inclined the P (31% and 48%), Fe (64% and 62%), K (34% and 100%), and Zn (156% and 188%) contents in roots and shoots, respectively, as compared with control treatment. The application of zinc–lysine (2.0 mM) improved the content of Zn (%) and decreased that of Na (%) in grains as compared with control, whereas the highest improvement was observed with the combined application of zinc–lysine (2mM) and biochar as it increased the Zn content (mg kg^-1^ of dry weight) and decreased the Na content (mg kg^-1^ of dry weight) in grains (**Figure 5**).

**Figure 5:** Data represented different levels of zinc-lysine (Control 0, 1, 2 mM) along with and without biochar on P in shoot, P in root, Fe in 638 root, Fe in shoot, K in root, K in shoot, Na in root, Na in shoot, Zn in root, Zn in shoot, Zn in grain, Na in grain of wheat plant showed means 639 of replicates (n=3) ± standard deviation. Different letters indicate significant differences by Tukey HSD test at p ≤ 0.05.

## Discussion

Salinity is one of the major threats to global food security levels amongst the much serious environment stressors which reduce the crop yield production. According to the previous studies that at the lateral stages of plant growth and lessening crop yield due to the salt stress negatively effect on the growth and reduce various biochemical, physiological and metabolic processes at the lateral stages of plant growth, lessening crop yield (Singh et al., 2014; Akhtar et al., 2015a; Kaya et al., 2020; Zafar et al., 2021; Ali et al., 2022). The present study was conducted for the impact estimation of salinity stress on different morphological, physiological, and biochemical attributes of wheat and the role of Zn–lysine alone or in combination with biochar. The lowest values of the physiological parameters such as chlorophyll a, b, total chlorophyll, carotenoids, *Pn*, *gs*, *Tr*, and *WUE* were observed in control plants (**Figure 2**). The salinity stress reduced the plant growth and crop yield by disrupting various physiological (*Pn*, *gs*, *Tr*, and *WUE*) and biochemical processes (oxidants and antioxidants) similar to our study (Emam et al., 2013; Kamran et al., 2019; Yadav et al., 2020). Our results about physiological attributes such as chlorophyll a, b, total chlorophyll, carotenoids, *Pn*, *gs*, *Tr*, and *WUE* are similar to previous studies which state that salt stress decreased these attributes and biochar and zinc–lysine enhanced these attributes (Sohi et al., 2010; Sahin et al., 2018; Parkash and Singh, 2020; Ali et al., 2021a; Ali et al., 2022). To promote better crop development for increased biomass and agricultural output, oxidative damage in response to salt stress may cause severe damage to photosynthetic pigments (chlorophyll and carotenoids), which can have a significant impact on radiation interception and water use efficiency by the crop canopy (Ali et al., 2021b).

Likewise, the processes are necessary for healthy growth in the salt stressed condition like essential physiological and biochemical disrupting and severe damage of cellular by excessive generation of reactive oxygen species (Saleem et al., 2020; Ghafar et al., 2021; Hameed et al., 2021; Perveen et al., 2021). The largest cellular generation of ROS, particularly H_2_O_2_, promoted lipid peroxidation of cellular membranes (Kazemi et al., 2019; Saleem et al., 2020), resulting in the synthesis of higher MDA in plant tissues in the current study. The output of the above literature is similar to our study showing that salt stress enhanced the accumulation of excessive salt ions in plant cells beyond the threshold limit which may cause cell damage and generate ROS species resulting in increased levels of MDA, H_2_O_2_, and EC (**Figure 3**). Induced irreversible damage to cellular membrane, resulting in increased electrolyte leakage at times of extreme stress by increase the accumulation of salt (Chantre Nongpiur et al., 2016). Numerous studies found that oxidant activity was regulated in maize (Lashari et al., 2015) with biochar application in salt-affected soil, wheat, and rice with Zn–lysine (Ali et al., 2022) and in eggplant with application of biochar (Parkash and Singh, 2020). A similar trend was observed in our results that MDA, H_2_O_2_, and EL were increased under salt stress but were decreased under Zn–lysine and biochar treatments (**Figure 3**). Improved and positive activities of antioxidant enzymes determined by the level of salt tolerance in the plants (Farhangi-Abriz and Torabian, 2018; Chen et al., 2020). Cai et al. (2019) found that salt tolerant cultivars have higher enzyme activity and related gene expression than moderately tolerant and salt-sensitive plants. Soil salinity decreased the antioxidant activity in borage plants, and application of biochar enhanced SOD, POD, and CAT activities (Farouk and AL-Huqail, 2022), as well as in jute (*Corchorus olitorius* L.) (Hasanuzzaman et al., 2017); the above findings support our study that the combined application of zinc–lysine and biochar statistically enhanced the POD, SOD, APX, and CAT activities under salt stress, as shown in **Figure 3**. So, in the salt affected soils are zinc application could abate possible Na^+^ and Cl^–^ in juries such as ROS production and lipid peroxidation in the plant by Zinc has regulatory role the Na^+^ and Cl^–^ uptake and translocation rate. The decrease in H_2_O_2_ was achieved upon Zn supplementation to seedlings growing with salt (Al-Zahrani et al., 2021).

The lowest values of growth attributes such as shoot length, root and shoot fresh and dry weights, grain weight, and spike length were observed in control plants (**Figure 4**). It was found that application of biochar alone enhanced the root, shoot growth and yield of eggplant (Parkash and Singh, 2020), and grain yield of wheat (El-sayed et al., 2021; Ali et al., 2021a) and zinc–lysine alone increased the growth parameters of wheat and rice such as root and shoot length, root and shoot fresh and dry weights, grain weight, and spike length (Ali et al., 2021b; Ali et al., 2022). The results of our study are in line with the above studies that biochar and zinc–lysine alleviate salinity stress in wheat plants.

Salinity stress caused the accumulation of salts (Na^+^, K^+^, Cl^+^) beyond the threshold limits in the maize plant rhizosphere (AbdElgawad et al., 2016). Results are in line with the above studies that excessive uptake of sodium ions (Na^+^) is found in roots, shoots, and grains. Furthermore, the application of zinc–lysine enhanced the P, Fe, K, and Zn concentrations in roots, shoots, and grains of wheat as compared with control, as described in other studies (Mobeen et al., 2021; Saleem et al., 2021). The application of biochar decreased Na^+^ in roots and shoots (Farouk and AL-Huqail, 2022). Plants have the ability to maintain an optimal K^+^: Na^+^ ratio in the cytosol, which impacts their ability to survive in saline circumstances (Mobeen et al., 2021; Saleem et al., 2021). The results of this study showed that overall wheat growth, physiology, nutrient uptake, and oxidant and antioxidant enzyme activity were regulated with zinc–lysine and biochar application.

## Conclusion

The present study investigated in the wheat plant the effect of the abiotic effect salinity stress on biochemical attributes, numerous growth and physiological attributes and alleviating potential of biochar in combination with zinc–lysine. It was observed that the soil salinity resulted in lower plant growth and yield of wheat. Contrarily, the application of Zn–lysine alone or combined with biochar enhanced the plant growth by alleviating the toxic effect of salinity and most likely by increasing antioxidant enzyme activities. It was concluded that the combined application of Zn–lysine and biochar improved the growth and physiology, and it may be the best combination to improve the grain quality of wheat plants under moderate salinity. However, studies that many other plant species in various concentrations salt stress are required for the better understanding the alleviating action of combine application of biochar and zinc-lysine under salt stress.

## Data availability statement

The original contributions presented in the study are included in the article/supplementary material. Further inquiries can be directed to the corresponding author.

## Author contributions

SAl: supervision, resources, funding acquisition, formal analysis, investigation, writing—original draft, writing—review and editing. ZA and WO: formal analysis, investigation, statistical analyses, writing—original draft, writing—review and editing. MN and MA: resources, data curation, methodology, software. MR and DD: project administration, methodology, formal analysis, writing—original draft, writing—review and editing. SAh and AA: writing—review and editing, writing—original draft, writing—review and editing. All authors contributed to the article and approved the submitted version.
